The article "Emulsions Made of Oils from Seeds of GM Flax Protect V79 Cells against Oxidative Stress" was published in 2015. Journal: Oxid Med Cell Longev.

# Emulsions Made of Oils from Seeds of GM Flax Protect V79 Cells against Oxidative Stress

**DOI:** 10.1155/2016/7510759

**Published:** 2015-12-08

**Authors:** Katarzyna Skorkowska-Telichowska, Karolina Hasiewicz-Derkacz, Tomasz Gębarowski, Anna Kulma, Helena Moreira, Kamil Kostyn, Katarzyna Gębczak, Anna Szyjka, Wioleta Wojtasik, Kazimierz Gąsiorowski

**Affiliations:** ^1^Department of Endocrinology, 4th Clinical Military Hospital, Rudolfa Weigla 5, 50-981 Wrocław, Poland; ^2^Faculty of Biotechnology, University of Wrocław, Przybyszewskiego 63/77, 51-148 Wrocław, Poland; ^3^Department of Basic Medical Sciences, Wrocław Medical University, Borowska 211, 50-556 Wrocław, Poland

## Abstract

Polyunsaturated fatty acids, sterols, and hydrophilic phenolic compounds are components of flax oil that act as antioxidants. We investigated the impact of flax oil from transgenic flax in the form of emulsions on stressed Chinese hamster pulmonary fibroblasts. We found that the emulsions protect V79 cells against the H_2_O_2_ and the effect is dose dependent. They reduced the level of intracellular reactive oxygen species and protected genomic DNA against damage. The rate of cell proliferation increased upon treatment with the emulsions at a low concentration, while at a high concentration it decreased significantly, accompanied by increased frequency of apoptotic cell death. Expression analysis of selected genes revealed the upregulatory impact of the emulsions on the histones, acetylases, and deacetylases. Expression of apoptotic, proinflammatory, and anti-inflammatory genes was also altered. It is thus suggested that flax oil emulsions might be useful as a basis for biomedical products that actively protect cells against inflammation and degeneration. The beneficial effect on fibroblast resistance to oxidative damage was superior in the emulsion made of oil from transgenic plants which was correlated with the quantity of antioxidants and squalene. The emulsions from transgenic flax are promising candidates for skin protection against oxidative damage.

## 1. Introduction

Reactive oxygen species (ROS) and reactive nitrogen species (RNS, e.g., nitric oxide, ^•^NO) are well recognized for playing a dual role as being both deleterious and beneficial [1]. At low to moderate concentrations they play physiological role in all cells, including defence against infectious agents and a number of cellular signalling pathways that regulate protein modification, gene expression, cell proliferation, migration and differentiation, and tissue remodelling [2]. However, overproduction of ROS or insufficiency of cellular antioxidative systems leads to oxidative damage and inhibits the normal functions of lipids, proteins, and DNA. Such states are major contributors to aging and the degenerative diseases such as chronic wounds, cancer, cardiovascular disease, hypertension, diabetes mellitus, immune system decline, and brain dysfunction [1, 3, 4]. Various environmental stresses induce excessive production of ROS that triggers cellular senescence and abnormal differentiation. The antioxidant systems in the cell can scavenge ROS and prevent irreversible cellular oxidative damage under normal conditions. However, there are instances where ROS production exceeds cell capacity for ROS scavenging. This situation can occur, for example, after UV irradiation or chemotherapy. The cells capacity to neutralize free radicals also decreases with age [5]. Therefore the use of antioxidant supplements as a defensive approach against cell damage caused by oxidative stress has been suggested. It was shown that the use of mixture of synergistic antioxidants is a good strategy providing better results than single components [6]. Oil obtained from flax (*Linum usitatissimum* L.) seeds is one of such natural preparations which could be used for prevention of oxidative cell damage. Flax oil contains high quantities of biologically active compounds such as unsaturated fatty acids (mostly *α*-linolenic acid and linoleic acid) and several components from isoprenoid pathway, such as squalene [7], phytosterols (mostly campesterol, stigmasterol, and *β*-sitosterol) [8, 9], carotenoids (lutein), and tocochromanols (tocopherols and plastochromanol-8) [10–12] and squalene, with anti-inflammatory properties. An exceptional group of oil constituents is polyphenols, which are the strongest free radical scavengers; they act directly or in a series of coupled reactions with antioxidant enzymes. They have the capacity to reduce DNA damage and prevent carcinogenesis, mainly by preventing deleterious actions of reactive oxygen species [13]. Although highly beneficial, the level of phenolic components in natural flax oil is quite low. Therefore, in order to enhance the antioxidant capacity of flax oil and by extension its stability, three types of GM flax plant with increased content of phenolic components in seeds were developed. In the first type of flax, the chalcone synthase gene was suppressed through the plant's transformation with a homologous gene construct (W86 line) [14]. In the second type, a triple-gene construct was introduced into the flax genome, which contained heterologous chalcone synthase, chalcone isomerase, and 4-dihydroflavonol reductase (W92 line) genes in the sense orientation [15], and, in the third type, the heterologous, sense-oriented O-glucosyltransferase gene, specific for flavonoid glycosylation and thus affecting flavonoids' stability, was introduced (GT line) [16]. As a result, the oil from transgenic flax types contained an increased level of cinnamic acid derivatives such as p-coumaric, caffeic, ferulic, and chlorogenic acids; vanillin, syringic, and coniferyl aldehyde; and flavonoids (kaempferol, luteolin, and apigenin) in varying proportions, but all of them were more stable than oil from wild-type flax [17, 18]. One of the oils was previously successfully used as a supplementation of wound healing regimen based on flax fabric providing unsaturated fatty acids and antioxidants that increased wound healing rate [19]. So it was believed that such oil can be good basis for a preparation protecting cells from oxidative damage. The purpose of this study was to estimate the impact of emulsions made of oils obtained from seeds of GM flax plants on Chinese hamster lung fibroblast (V79) proliferation, frequency of apoptosis and necrosis, content of intracellular free oxygen radicals, the level of DNA strand breaks, and expression level of selected genes connected with apoptosis, inflammation, and histone modification. V79 cells were chosen as they are often applied in studies on cytotoxic and genotoxic effects of oxidative stress, because of genetic alterations which make these cells more sensitive to oxidative damage; for instance, the antioxidant enzyme heme oxygenase-1 is not inducible in V79 cells during the adaptive response to oxidative stress [20].

The article "Emulsions Made of Oils from Seeds of GM Flax Protect V79 Cells against Oxidative Stress" was published in 2015. Journal: Oxid Med Cell Longev.

## 2. Materials and Methods

### 2.1. Plant Material

Transgenic flax plants were obtained by agrotransformation of the* Linum usitatissimum* L. cv. Linola. The W92 line was generated using a binary vector with three gene constructs containing cDNAs encoding chalcone synthase (CHS, EMBL/GenBank database access number X04080), chalcone isomerase (CHI, EMBL/GenBank database access number X14589), and dihydroflavonol 4-reductase (DFR, EMBL/GenBank database access number X15537) from* Petunia hybrida* in the sense orientation and under the control of the strong and nonspecific 35S CaMV promoter and OCS terminator [21]. In W86, repression of the endogenous chalcone synthase gene was achieved by overexpression of cDNA of the* P. hybrida* homologue (CHS, EMBL/GenBank database access number X04080), via the siRNA mechanism [14]. The GT transgenic plants were obtained using the construct containing the 7-O-glycosyltransferase gene (SsGT1, EMBL/GenBank database accession number AY033489) derived from* Solanum sogarandinum* in the sense orientation under the control of the seed-specific NAP (napin) promoter and OCS terminator [18]. Seeds from the fifth generation of field-grown transgenic plants (W92, W86, and GT types) from the 2012 vegetative season were used as an oil source throughout this study. Preparation of oil from flax seeds and emulsion made of oil followed the procedures previously described [14].

The article "Emulsions Made of Oils from Seeds of GM Flax Protect V79 Cells against Oxidative Stress" was published in 2015. Journal: Oxid Med Cell Longev.

### 2.2. Fatty Acid Content in Oil from Flax Seeds

Fatty acid methyl esters were prepared in accordance with the method previously described [22] and analyzed by means of gas chromatography [23]. Trimethylsilyl derivatives of sterols were prepared [24] and analyzed with a 6890 N gas chromatograph equipped with an FID detector and the capillary column HP-5 30 m × 0.32 mm × 0.25 *μ*m (Agilent Technologies, USA) using helium as a gas carrier, 5*α*-cholestane as an internal standard for quantitative analysis, and Chemstation v. B.04.02 for calculation of the results.

### 2.3. GC-FID Analysis of Squalene and Sterols

1 mL of oil was extracted twice with 10 mL of hexane by vortexing vigorously for 15 min. The extracts were pooled and evaporated under nitrogen (25°C) to dryness. Trimethylsilyl derivatives of sterols were prepared according to the method described by Shukla et al. [24]. The separation of silyl compounds and the quantification were performed on a gas chromatograph 6890 N (Agilent Technologies, USA) equipped with an FID detector and the capillary column HP-5 30 m × 0.32 mm × 0.25 *μ*m (Agilent Technologies, USA). Helium was used as a carrier gas at a flow rate of 1.0 mL/min and the separation was carried out at a temperature set from 250°C (for 5 min) to 290°C (for 14 min); the temperature increased at a rate of 5°C/min. 5*α*-cholestane was used as an internal standard for quantitative analysis and Chemstation v. B.04.02 was used to calculate the results.

### 2.4. UPLC-PDA Phenolic and Terpenoid Components of Oil

The identification and quantification of components were done as described previously [20]. Methanol- and water-extracted compounds from the oil were measured using UPLC combined with two detectors (PDA and MS). The extracts from flax seed oil were analyzed in the Waters Acquity UPLC System with a 2996 PDA detector and Waters Xevo QTof MS System mass spectrometer, using an Acquity UPLC column BEH C18, 2.1 × 100 mm, 1.7 *μ*m.

The contents of lipid-soluble compounds were determined using a Waters Acquity UPLC System with a 2996 PDA detector. A sample of flax seed oil was dissolved with acetone, vortexed, and left at 4°C. Next, the samples were dissolved with a mixture of acetonitrile/methanol (1 : 1) and shaken for 1 min. This solution was directly injected onto a UPLC BEH C18, 2.1 × 100 mm, 1.7 *μ*m column after filtration through an Acrodisc 0.22 *μ*m filter (Gelman Sciences, Ann Arbor, MI). The identity of components was confirmed using authentic standards. The calculations were done after integration of peaks at maximum of the absorption for each component (e.g., 280 or 320 nm for phenolic acids, 290 nm for tocopherol, 350 nm for flavonoids, and 445 nm for lutein) against standard curves.

The article "Emulsions Made of Oils from Seeds of GM Flax Protect V79 Cells against Oxidative Stress" was published in 2015. Journal: Oxid Med Cell Longev.

### 2.5. Preparation of Oil Emulsions

Flax oil emulsion was prepared as described previously [25]. Briefly, soybean lecithin (Lipoid S75 from Lipoid, Ludwigshafen, Germany) and Tween 80 (Sigma-Aldrich, St. Louis, MO, USA) were mixed with flax oil, and then an aqueous phase containing glycerol (Sigma-Aldrich) was added. The oil and aqueous phases were mixed vigorously. The sample was further sonicated using a Microson ultrasonic cell disruptor (Misonix Inc., Farmingdale, NY, USA) for 10 min at 4 W. The sonicated preparations were filtered through sterile Acrodisc (Gelman Sciences, Ann Arbor, MI) 0.22 mm filters. All the emulsion samples were prepared at room temperature. The final concentrations of the chemicals in emulsion were 1% lecithin, 2.5% flax oil, 2.5% Tween 80, and 2.5% glycerol.

### 2.6. Cell Culture Media and Reagents

Cell culture media and reagents were obtained from Lonza (Verviers, Belgium). Plastic cell culture flasks and polystyrene culture plates were purchased from BD Bioscience (Bedford, MA, USA). The fluorochrome mixture, Alexa Fluor 488 AnnexinV/Dead Cell Apoptosis Kit, was from Invitrogen/Molecular Probes (Carlsbad, CA, USA). All other compounds used in the tests were from Sigma-Aldrich (St. Louis, MO, USA).

### 2.7. Cells and Culture Conditions

The Chinese hamster pulmonary fibroblasts (V79-379A cells) were obtained from the Institute of Immunology and Experimental Therapy of the Polish Academy of Sciences in Wroclaw, Poland. Cells were grown in EMEM with 2 mM L-glutamine, 10% FBS, and antibiotics: 100 U/mL penicillin and 0.1 mg/mL streptomycin, at 37°C in a CO_2_ incubator. On the day of the experiment, adherent cells were detached from culture plates with trypsin/EDTA solution, washed with PBS, and inspected for cell viability under a microscope after staining with a 0.4% solution of trypan blue, and cells were plated on 24-well plastic culture plates at initial cell densities of 1.5 × 10^5^ cells per well. After 24 h of culture at 37°C in the CO_2_ incubator, the oil emulsions were added to V79 cell cultures to the final concentrations of 0.5%, 1%, and 5% v/v, and incubation was continued for 48 h. The tested emulsions contain phenolic compounds, which could exert their antioxidative action both by direct scavenging of free radicals and by enhancing expression of endogenous antioxidative enzymes; thus such period of incubation is appropriate for evaluation of increased expression of antioxidative enzymes [26]. Where indicated, the cells were exposed to oxidative stress, resuspended with buffered saline without Ca^2+^ and Mg^2+^ ions, and incubated with hydrogen peroxide (100 *μ*M, 30 min, 4°C). Then, cells were washed with PBS and assayed for resistance to oxidative stress.

The article "Emulsions Made of Oils from Seeds of GM Flax Protect V79 Cells against Oxidative Stress" was published in 2015. Journal: Oxid Med Cell Longev.

### 2.8. Assessment of Cell Proliferation

After 48-hour incubation with the oil emulsions, V79 cell cultures were examined for cell density/cell proliferation with sulforhodamine B (SRB) and colorimetric measurement [27]. The absorbance of the SRB solution was estimated at *λ* = 540 nm in Victor 2 microplate reader (PerkinElmer, MA, USA).

### 2.9. Evaluation of Intracellular ROS Level

The cell-permeable, fluorescence probe DCFH-DA (2′7′-dichlorodihydrofluorescein diacetate, final concentration of 25 *μ*M) was added to the cell culture for the last 2 h of culture in the dark at 37°C in the CO_2_ incubator, according to the standard procedure [28]. Then, the cells were washed twice with PBS and treated with H_2_O_2_ (100 *μ*M) for 30 min. Fluorescence of dichlorodihydrofluorescein was measured (*λ*_ex._ = 485 nm, *λ*_em._ = 535 nm) in Victor 2 microspectrophotometer (PerkinElmer, Waltham, MA, USA). The applied concentration of H_2_O_2_ (100 *μ*M) was within the range of levels naturally present in skin wounds (50–200 *μ*M) [29]. Thirty-minute cell incubation with H_2_O_2_ was chosen, as data found in the literature strongly suggest that cells were able to decompose almost all the H_2_O_2_ in culture medium by 30 min [30].

### 2.10. Detection of Apoptosis and Necrosis

For detection of apoptosis and necrosis V79 cells were detached from culture plates with the trypsin/EDTA solution, washed with PBS, spun down, and stained with a mixture of fluorochromes (Alexa Fluor 488 AnnexinV and PI) according to the instructions of the manufacturer (Invitrogen/Molecular Probes, Carlsbad, CA, USA). After 15 min of incubation at room temperature in the dark, samples were acquired on a CyFlow Cube8 flow cytometer (Partec, Germany) and the fluorescence emission was measured using a 488 nm excitation laser lamp and 536/40 (BP) and 630 nm (LP) emission filters. The samples were analyzed with CyView software. Granulation, size, and fluorescence intensity were recorded for 40,000–100,000 cells. Percentages of viable, apoptotic, and necrotic (dead) cells were calculated from dot-plot graphs.

### 2.11. Analysis of DNA Damage by Comet Assay

Alkaline single-cell gel electrophoresis (comet assay) was carried out according to the routine procedure with minor modification [31]. The V79 cell suspensions were mixed with an equal volume of 1% low melting point agarose (Sigma type VII) at 37°C, transferred onto glass slides precoated with 0.5% of regular agarose (Sigma type I-A), and placed on ice for 5 min to solidify the agarose. Further procedures of cell lysis, relaxation of the DNA loops, and electrophoresis followed those described previously [32]. Finally, slides stained with the fluorescent dye (DAPI, 1 *μ*g/mL) were evaluated under a fluorescence microscope (Nikon Eclipse E-600) equipped with a Nikon UV 1A filter block and with the digital camera and computer with the CometPlus 2.5 software (Theta System Electronics GmbH, Gr$\ddot{o}$benzell, Germany). Seventy-five comets randomly found on each slide under a microscope were scored and the DNA content in the comet's head (%) and the Olive tail moment (OTM, arbitrary units) were analyzed.

The article "Emulsions Made of Oils from Seeds of GM Flax Protect V79 Cells against Oxidative Stress" was published in 2015. Journal: Oxid Med Cell Longev.

### 2.12. Expression Analysis of Selected Genes

The V79 cells pretreated for 48 hours with 0.5% oil emulsion were submitted to 100 *μ*M H_2_O_2_ treatment for 30 min. As a control, cells incubated without oil emulsion were used. The cells detached from culture wells were spun out, washed, and subjected to gene expression analysis. Total RNA was isolated from freshly harvested cells using an RNeasy Plus Mini Kit (Qiagen, Germany) according to the manufacturer's instructions. To eliminate any genomic DNA contamination, 2 *μ*g of each isolated RNA sample was treated with DNase I (Fermentas, Lithuania) and directly used as a template for cDNA synthesis. The cDNAs were synthesized using a High-Capacity cDNA Reverse Transcription Kit (Applied Biosystems, USA). Real-Time PCR reactions were set according to the SYBR Green Master Mix (Applied Biosystems, USA) producer's instructions; the primer sequences are presented in Table 1. Obtained data were analyzed using ΔΔCt methodology for calculation of the parameter RQ (relative quantification).

### 2.13. Statistical Analysis

The statistical significance of the results was assessed with the *t*-test for independent samples and with the two-way ANOVA.

## 3. Results

In order to detect their impact of emulsions based on oils from transgenic flax on alleviation of oxidative stress in V79 cells, several parameters were measured upon cell treatment.

### 3.1. Cell Proliferation and Antioxidative Status

Oil emulsions enhanced the proliferation and increased the number of V79 cells upon incubation (48 h) with low concentrations of oil emulsion (0.5%, 1% v/v). However, at high concentration (5% v/v), inhibition of cell proliferation and a decrease in the number of cells were observed. The respective data are presented in Figure 1. There is a significant difference in the activity of oil derived from two transgenic plant types. The emulsion based on oil from W86 flax seeds increased the V79 cell number by about 40% at concentration of 0.5% v/v, while oil emulsion from W92 seed increased the cell number by 30% as compared to the oil emulsion from seed of the control plant. In the case of the third analyzed transgenic plant type (GT) as well as the control nontransformed plant, the impact of oil emulsion on V79 cell proliferation was very slight and not significant.

The article "Emulsions Made of Oils from Seeds of GM Flax Protect V79 Cells against Oxidative Stress" was published in 2015. Journal: Oxid Med Cell Longev.

At high concentration (5%, v/v), all tested oil emulsions inhibited cell proliferation and reduced the cell number by about 25%. All the results were statistically significant.

Incubation of the cells with oil emulsions led to the significant reduction of intracellular ROS formation in cultures exposed subsequently to H_2_O_2_ (100 *μ*M for 30 min, at 4°C), as estimated with the DCFH-DA assay (Figure 2).

The decrease of intracellular ROS level was the highest in cultures incubated with W92 and W86 oil emulsions. The cellular ROS level was diminished by about 30% after treatment with the emulsion at the concentration of 0.5% and by 40% at the concentration of 5%. In the other two cases, where cells were incubated with the emulsion with oil from GT and Linola seeds, the intracellular ROS level was also reduced as compared to the control cultures (without oil emulsion), but the reduction was not significant.

### 3.2. Genomic DNA Analysis

Since oil emulsion reduces the intracellular ROS level, the genomic DNA protection against H_2_O_2_ damage was expected. Thus, we estimated the impact of oil emulsions on the level of DNA damage in V79 cell culture treated with hydrogen peroxide (data presented in Figure 3).

When compared to the control, each of the used emulsions significantly reduced the level of genomic DNA strand breaks caused by H_2_O_2_ as detected by the increased content of the DNA in comets' heads (by about 25% and 35% at the lowest and the highest oil emulsion concentration, resp.). Marked decreases of DNA level in the tail moment (damaged form) by about 44% and 56% in the lowest and the highest oil emulsion concentrations, respectively, were also detected. All these results (Figure 3) differed significantly from those for the control culture (untreated cells) as calculated with the *t*-test for independent samples.

It should be noted that, in the V79 cells incubated with the oil emulsion and not H_2_O_2_ treated, the level of DNA damage was insignificant. Moreover, the impact of various concentrations of oil emulsion on the DNA damage was not significant (data not presented in figures).

### 3.3. Cell Apoptosis

The frequency of occurrence of apoptotic and necrotic cells upon oxidative stress was measured (Figure 4). The V79 cell cultures incubated with the oil emulsions were treated with H_2_O_2_ (100 *μ*M) at 4°C for 30 min. For the control, cells were H_2_O_2_-treated without incubation with the oil emulsion.

The article "Emulsions Made of Oils from Seeds of GM Flax Protect V79 Cells against Oxidative Stress" was published in 2015. Journal: Oxid Med Cell Longev.

Transgenic flax oil emulsions (W92, W86, and GT) at 0.5% concentration had similar effect on apoptosis of the V79 cells and decreased it by 40–50%, whereas treatment with 5% oil emulsions led to an increase in the number of apoptotic cells by about 65%. In the case of the control oil emulsion (prepared from nontransgenic flax oil), low concentrations of the emulsion (0.5% and 1%) did not affect the frequency of apoptotic cells, whereas at the concentration of 5% a marked increase of apoptotic cell number (by about 75%) in comparison to the control culture (without oil emulsion) was observed. The two-way ANOVA test proved that differences in the frequency of apoptotic cells treated with H_2_O_2_ between the tested emulsions were insignificant (*p* = 0.113), while the impact of various concentrations of emulsions was highly significant (*p* < 10^−4^). The frequency of cells exhibiting necrosis upon H_2_O_2_ treatment was reduced by about 70–80% when cells preincubated with each of the oil emulsions were compared to control cultures (cells treated with H_2_O_2_ without preincubation with oil emulsion). Two-way ANOVA showed that differences in the frequency of necrotic cells in cultures preincubated with all three oil emulsions were insignificant (*p* = 0.229) and also the concentration of oil emulsion does not significantly affect the frequency of necrotic cells (*p* = 0.737).

In summary, it should be pointed out that all three oil emulsions protect V79 cells against oxidative stress at low concentrations, while at high concentration they promote apoptotic cell death.

### 3.4. Constituents of Oil Emulsion

The content of compounds in four types of oil emulsions is presented in Table 2. The compounds were identified and estimated with the UPLC method for phenolics and terpenoids [20] and with GC-FID for sterols and fatty acids; then the results were summed up to give the total contents in the assigned group of compounds: lipid-soluble antioxidants, phenolics, unsaturated fatty acids, squalene, and sterols.

The content of lipid-soluble antioxidants (lutein, *γ*-tocopherol, and plastochromanol-8) in W86 and W92 oil emulsions was higher than in oil emulsion from nontransgenic flax seed (Linola) by 23% and 20%, respectively, while GT oil emulsion contains a lower (by 15%) quantity of these compounds compared to control seed oil emulsion.

The total contents of phenolics (ferulic acid, coumaric acid, caffeic acid, cinnamic acid, chlorogenic acid, syringic aldehyde, and vanillin) in oil emulsions from transgenic flax plants were 2-3 times higher than in the Linola oil emulsion, being the highest in the W86 oil emulsion. A significant increase in the squalene level was noted for both the W92 and W86 oil emulsions; the content of this compound was almost 3 times higher than in oil emulsion from GT and the control plants. The content of unsaturated fatty acids (oleic acid, linoleic acid, and *α*-linolenic acid) and sterols (campesterol, stigmasterol, *β*-sitosterol, and cycloartenol) was quite similar in the oil emulsions from transgenic flax plants (W92, W86, and GT) and from the nontransgenic plant (Linola). The detailed analysis of fatty acids, tocochromanols, carotenoids, and phenolics in those oils was published previously [20].

The article "Emulsions Made of Oils from Seeds of GM Flax Protect V79 Cells against Oxidative Stress" was published in 2015. Journal: Oxid Med Cell Longev.

### 3.5. Expression of Selected Genes

Flax oil contains several secondary metabolites originating from the phenylpropanoid and isoprenoid pathways. These compounds revealed strong antioxidant activity and thus may strengthen anti-inflammatory properties of oil emulsions. In order to analyze the oil emulsion's impact on V79 cell physiology, expression of selected genes was investigated. Cells not treated with oil emulsion served as a control.

Numbers of essential cellular processes such as gene regulation, DNA damage response, gene dosage compensation, and cell viability are regulated by histone and nonhistone proteins' modification. Acetylation of histone is now recognized as a key regulator of chromatin activity [33] and thus expression of genes coding for acetylases and deacetylases was investigated. In all cases the reasonable induction of MYST1 and MYST2 genes' expression was detected (Figure 5(a)). Only a slight reduction of HAT1 acetylase gene expression was found.

The central regulators of apoptotic cell death are BCL2 gene family members (Bcl-2, Bcl-xl, Bax, and Bak). The loss of their function caused necrotic cell death. Each of four oil emulsions activated all analyzed genes, the strongest activation being observed for Bcl-2 and Bax (Figure 5(b)). The result of proapoptotic gene analysis is interesting. Stimulation of CASP9 gene expression was detected upon cell treatment with all oil emulsions. It is known that CASP8 enzyme activates sequentially other family members, CASP9 and CASP3 among them. These downstream enzymes play the central role in the execution phase of cell apoptosis. However, in no case was the CASP8 and CASP3 gene expression affected. Strong activation of the gene coding for DNA fragmentation factor (DFF) was recorded. In mammalian cells DFF enzyme is activated by caspase-3 cleaving.

The article "Emulsions Made of Oils from Seeds of GM Flax Protect V79 Cells against Oxidative Stress" was published in 2015. Journal: Oxid Med Cell Longev.

Since oil emulsion constituents reveal high antioxidant capacity, the selected genes involved in the inflammatory response of treated V79 cells were analyzed (Figure 5(c)). The data obtained strongly suggest the positive impact of all oil emulsions on the expression level of proinflammatory IL-6 and anti-inflammatory ICAM genes. In all four cases the level of IL-6 cytokine was reduced at least threefold as compared to the control cells. The anti-inflammatory ICAM gene expression level was increased compared to control untreated cells.

## 4. Discussion

Reactive free radicals promote cell apoptosis by impairing numerous cellular mechanisms. It was shown that oxidative stress promotes damage to many cellular mechanisms and causes fibroblast apoptosis [34]. It is already well evidenced that small molecules from plant secondary metabolism act as scavengers of radicals and thus protect the cell against damage. For example, it was shown that low molecular phenylpropanoids such as phenolic acids, flavonoids, and many others act as strong antioxidants [35–37]. It was also reported that low-molecular-weight antioxidative compounds originating from the phenylpropanoid pathway can protect the skin cells from oxidative damage [38, 39]. The important aspect is that they exert their beneficial effects by acting as chain-breaking antioxidants, inhibiting lipid peroxidation of polyunsaturated fatty acids contained within biological membranes, thereby preventing the formation of potentially cytotoxic and highly reactive aldehydes. This was the reason to exploit oils obtained from genetically engineered plants producing higher levels of phenylpropanoids for cell protection against oxidative injury. Our reasoning for use of flax oil instead of a plant extract was that also other constituents of oil can display protective properties. For example, squalene as an antioxidative compound protects cellular and cytoplasmic biomembranes from oxidative stress [40]. Sterols, although weak antioxidants [41], are considered as lipid agents protecting against oxidation [42, 43]. Flax oil is a rich source of omega-3 and omega-6 fatty acids that has been reported as having a beneficial influence on wound healing [44]. The polyunsaturated fatty acids (PUFAs) are known to be involved in scavenging hydroxyl radicals, forming hydroxyl-fatty acids as a product [45]. It is thus suggested that all these oil emulsion constituents may help to reestablish the redox balance by determining a chain reaction of oxidizing events. The important fact is that they act synergistically and a mixture of antioxidants is more efficient than a single type of antioxidant [46]. Thus, it was possible that supplying the cells with essential fatty acids and antioxidants can help strengthen the plasma membranes and combat oxidative stress in damaged tissues.

The article "Emulsions Made of Oils from Seeds of GM Flax Protect V79 Cells against Oxidative Stress" was published in 2015. Journal: Oxid Med Cell Longev.

Indeed, the positive effect of the emulsions prepared in three concentrations (0.5%, 1%, and 5%) from oils obtained from seeds of three transgenic flax types (W86, W92, and GT) on* in vitro* cultured Chinese hamster pulmonary fibroblasts (V79 cell line) was detected except where high concentration was used. Spearman's rank correlation between the antioxidant potential of the oil emulsions and the content of selected groups of active compounds showed that the level of phenolics and lipid-soluble antioxidants concomitant with squalene strongly correlates with the cells' resistance against oxidative stress (Table 3). At high concentration, apoptotic cell death significantly increases, cell proliferation decreases, and a slight increase in genomic DNA damage was detected. The reason for this is as yet unknown, but it is suggested that a high antioxidant concentration might promote prooxidative effects. This suggestion is supported by the finding that during oxidative stress polyphenols may act as prooxidants and may induce apoptosis and prevent tumour growth [47]. Also it was reported that polyunsaturated fatty acids at medium concentration cause apoptotic cell death, while at high concentration they induce cell necrosis [48]. It was documented that n-6 PUFAs such as *α*-linolenic acid inhibit expression of arachidonate-metabolizing enzymes (COX and LOX), resulting in accumulation of the nonesterified form of arachidonic acid. The elevated content of this compound form induces mitochondrial cytochrome C release and causes direct activation of caspase-3 [49, 50]. PUFAs of n-3 type are able to induce both extrinsic and intrinsic pathways of apoptosis, directly activating caspase-3, caspase-8, and caspase-9, increasing expression of the proapoptotic proteins Bak and Bcl-xS and reducing the antiapoptotic proteins Bcl-2 and Bcl-xL [50]. Certainly, we demonstrated the upregulatory effect of oil emulsions on the Bcl-2 gene family as well as on caspase-9 gene expression.

Detailed, multicriterial analysis (Table 4) indicates that the most effective in cell protection were W86 and W92 oil emulsions, while the efficiency of GT oil emulsion activity differs significantly from that of W86 and W92, although the total antioxidants level in all three oil emulsions is quite similar. The only components whose concentration was lower in GT than in W79 and W86 oils were p-coumaric acid and plastochromanol-8 [20]. This needs to be further investigated if those components are better able to protect cell from oxidative damage than other phenolic acids and terpenoids.

The article "Emulsions Made of Oils from Seeds of GM Flax Protect V79 Cells against Oxidative Stress" was published in 2015. Journal: Oxid Med Cell Longev.

However, the compound which differentiates the emulsions most strongly is squalene. Thus, it is suggested that although all antioxidants are involved in oil emulsion antioxidant potential, the squalene molecule produces a more efficient effect. Squalene is the main precursor of sterol, which controls membrane fluidity and permeability. Besides strong antioxidant activity, squalene is a potential immunologic adjuvant (called MF59) which stimulates the immune system when administered with a vaccine [51, 52]. Although the mechanism of action remains unknown, MF59 is capable of affecting the cell behaviour by changing the lipid metabolism, namely, by inducing accumulation of neutral lipids within the target cells [53]. More likely, however, MF59 is capable of switching on a number of genes. Induction of as many as 891 genes in mouse muscle has been detected. Most activated genes concern cytokines and cytokine receptors. Among them was a group of Ccl chemokines involved in inflammatory processes [52]. Although all antioxidative oil constituents protect cells against oxidative damage primarily through scavenging of free radicals, their mode of action might be far beyond this direct action [54, 55]. It might be considered that cells respond to antioxidants through direct interactions with enzymes involved in signal transduction; for instance, they may modulate activity of NF-*κ*B and glutathione biosynthesis, activate nuclear redox factor NRF2, and mediate activity of crucial enzymes of free radical pathways, such as NADPH oxidase, superoxide dismutase, xanthine oxidase, and 5-lipoxygenase [56]. For example, it was documented that *β*-sitosterol activates sphingomyelinases, which leads to an increase of ceramide and ceramide-dependent pathways of apoptosis. It also enhances expression of Fas protein, apoptosis inducing ligand (TRAIL) and directly activates caspase-8, thus inducing receptor-mediated apoptosis [41]. More likely, cells might respond to antioxidants through direct interactions with receptors and thus regulate chromatin activity and affect expression of selected genes. Activation of the histone acetyltransferase-deacetylase system, upregulation of genes involved in apoptotic cell death, and downregulation of proinflammatory gene expression suggest the active role of oil emulsion constituents in cell activity. Since the level of gene expression was independent of the oil's origin, the final impact is perhaps the result of synergy between oil constituents rather than their individual concentration. Perhaps induction of deacetylases (HD1, HD2, HD3, and HD8) in almost all cases strengthens the effect of acetylases. Thus the compounds that constitute flax oil emulsions are important players in chromatin activity of V79 cells, which might be beneficial when applied for skin wound healing.

The article "Emulsions Made of Oils from Seeds of GM Flax Protect V79 Cells against Oxidative Stress" was published in 2015. Journal: Oxid Med Cell Longev.

The data suggest that on one hand all four oil emulsions enable activation of the antiapoptotic programme but, on the other, they promote proapoptotic activity in treated cells. Thus it might be suggested that injured cells are directed to the apoptotic rather than the necrotic death programme when treated with oil emulsion. This is important for wound treatment since enzymes released from necrotic cells might cause damage of surrounding tissue.

In conclusion, the oil emulsions based on oil from transgenic flax seeds (W86, W92, and GT) are more effective than those from the control plants in relation to the fibroblasts' resistance to oxidative damage. The data suggest that W86 and W92 oil emulsions might be beneficial in skin protection against oxidative stress.

## Figures and Tables

**Figure 1:** Proliferation of the V79 cells after 48-hour incubation with the tested emulsions in three different concentrations (0.5%, 1%, and 5%). Results of the SRB spectrophotometric assay obtained with the tested emulsions are presented as *x*-fold of the control culture (cells excluding previous incubation with the tested emulsions; value = 1) and are means of 8 independent experiments ± SD. Statistical significance of differences between the results with the tested emulsions compared to those in the control cultures was calculated with *t*-test for independent samples (^*∗*^ *p* < 0.05, ^*∗∗*^ *p* < 0.01, and ^*∗∗∗*^ *p* < 0.001).

**Figure 2:** The contents of ROS in V79 cells cultured for 48 h with the presence of the tested emulsions in three different concentrations (0.5%, 1%, and 5%) and subsequently exposed to H_2_O_2_ (100 *μ*M, 30 min, 4°C). The results are presented as *x*-fold of the control culture (cells exposed to H_2_O_2_ excluding previous incubation with the tested emulsions; value = 1) and are means of 8 independent experiments ± SD. Statistical significance was calculated with *t*-test for independent samples (^*∗*^ *p* < 0.05, ^*∗∗*^ *p* < 0.01, and ^*∗∗∗*^ *p* < 0.001).

**Figure 3:** The influence of the tested emulsions in three different concentrations (0.5%, 1%, and 5%) on DNA damage in V79 cells exposed to H_2_O_2_ (100 *μ*M, 30 min, 40°C). The contents of DNA in the comets' heads (a) and the Olive tail moment (OTM) (b) were measured in 75 comets, randomly found under a fluorescence microscope. The control cultures (C) contained V79 cells incubated for 48 h without the tested emulsion and then exposed to H_2_O_2_. The results are presented as mean of 8 independent experiments ± SD. Statistical significance was calculated with *t*-test for independent samples (^*∗*^ *p* < 0.05, ^*∗∗*^ *p* < 0.01, and ^*∗∗∗*^ *p* < 0.001).

The article "Emulsions Made of Oils from Seeds of GM Flax Protect V79 Cells against Oxidative Stress" was published in 2015. Journal: Oxid Med Cell Longev.

**Figure 4:** The frequency of apoptosis (a) and necrosis (b) in V79 cell cultures exposed to oxidative stress (H_2_O_2_; 100 *μ*M, 30 min, 40°C) after 48-hour incubation with the tested emulsions in three different concentrations (0.5%, 1%, and 5%). Control cultures (C) contained V79 cells incubated for 48 h without the tested emulsion and then exposed to H_2_O_2_. The results are presented as mean of 8 independent experiments ± SD. ANOVA was used for statistical significance calculation (^*∗*^ *p* < 0.05 and ^*∗∗*^ *p* < 0.01).

**Figure 5:** Level of selected acetylase/deacetylase (a), apoptotic (b), and inflammation (c) gene expression. Cells incubated with the flax oil emulsion (0.5%) were harvested, RNA isolated, and converted to cDNA which served as a template for gene amplification using RT-PCR. Primers used are depicted in Table 1 in Section 2. mRNA from nontreated cells was used for control. Expression data were expressed as fold of control value (mean value of 3 independent experiments ± SD; control = 1).

**Table 1:** Primers used for detecting expression of selected genes in V79 cells.

*Cricetulus griseus* glyceraldehyde 3-phosphate dehydrogenase	
GAPDH_FP-GGCAAAGTCATCCCAGAG, GAPDH_RP-CTCAGATGCCTGCTTCAC	

*Cricetulus griseus* interleukin-6	
IL6_FP-AGCAAGAGTCATTCAGAGC, IL6_RP-GTTCGATGGTCTTGGTCC	

*Cricetulus griseus* intercellular adhesion molecule 1	
ICAM1_FP-CCATGAACGGTACCTACG, ICAM1_RP-TATCCTGATCTTTCTCTGGCG	

*Cricetulus griseus* histone acetyltransferase 1 (Hat1)	
HAT1_FP-ATGTAGAGGCTTTCGAGAATATC, HAT1_RP-GCAAAGAGCGTAGCTCC	

*Cricetulus griseus* K(lysine) acetyltransferase 7 (MYST2)	
MYST2_FP-TGTCCCACAGGCAAGAT, MYST2_RP-CCCGAGTGTTCCCATAG	

*Cricetulus griseus* K(lysine) acetyltransferase 8 (MYST1)	
MYST1_FP-CTATCGCAAGAGCAACATC, MYST1_RP-CCTTGCCTATCTACTTCCG	

*Cricetulus griseus* histone deacetylase 2 (Hdac2)	
HD2_FP-TCACTGTCTGGTGATAGGC, HD2_RP-ATATGTCCAACACCGAGC	

*Cricetulus griseus* histone deacetylase 3 (Hdac3)	
HD3_FP-GGTGGACTTCTACCAACC, HD3_RP-CCGGGCAACATTTCGGA	

*Cricetulus griseus* histone deacetylase 1 (Hdac1)	
HD1_FP-CCCTTCCAATATGACCAACC, HD1_RP-GTCTTCTTCATCCTCATCACC	

*Cricetulus griseus* histone deacetylase 8 (Hdac8)	
HD8_FP-ACTGATGGCTATCTGCAAC, HD8_RP-CAGCGGTGATTGTAGCTC	

*Cricetulus griseus* caspase-3	
Casp3_FP-AGGGAGACATTCATGCG, Casp3_RP-TCCTTCTTCACCATGGCT	

*Cricetulus griseus* caspase-8	
Casp8_FP-GGGAGAGTTACTTCAGAATGC, Casp8_RP-GGTATGTTCTTCCTCGCC	

*Cricetulus griseus* caspase-9	
Casp9_FP-CACCCTGGCTTCATTCTT, Casp9_RP-CTTCGATGGCTCCAACT	

*Cricetulus griseus* Bcl-2-associated X protein (Bax)	
Bax_FP-GGGTTTCATCCAGGATCG, Bax_RP-CTCTGCAGCTCCATGTT	

*Cricetulus griseus* Bcl-2 homologous antagonist killer (Bak)	
Bak_FP-CCTATTTAAGAGCGGCATCAG, Bak_RP-CGATGCAATGGTGCAGTA	

*Cricetulus griseus* Bcl-xL	
Bcl-xL_FP-TCAATGGCAACCCATCCT, Bcl-xL_RP-GTACCGCAGCTCAAACTC	

*Cricetulus griseus* B-cell CLL/lymphoma 2 (Bcl-2)	
Bcl-2_FP-GGGATTCCTACGGATTGAC, Bcl-2_RP-CAACGACACCATCGATCT	

The article "Emulsions Made of Oils from Seeds of GM Flax Protect V79 Cells against Oxidative Stress" was published in 2015. Journal: Oxid Med Cell Longev.

**Table 2:** The contents of the selected compounds in the tested emulsions from plants of three transgenic lines and a nontransgenic flax (Linola). The mean and standard deviation (SD) values obtained from analyses of oil samples were calculated for 1 mL of emulsion. The estimation of lipid-soluble antioxidants and phenolics was done by means of the UPLC method, while the fatty acid and sterols contents were determined by GC-FID.

Estimated compounds	Linola		W92		W86		GT	
	Mean; *n* = 3	SD	Mean; *n* = 3	SD	Mean; *n* = 3	SD	Mean; *n* = 3	SD
Lipid-soluble antioxidants [*μ*g/mL]	20.53	1.68	24.67	1.32	25.27	0.87	17.68	0.75
Phenolics [ng/mL]	1.05	0.24	1.88	0.44	3.20	0.34	2.28	0.32
Unsaturated fatty acids [mg/mL]	21.50	0.50	22.73	0.49	19.87	0.81	21.21	0.50
Squalene [*μ*g/mL]	1.83	0.20	5.37	0.31	4.96	0.34	1.94	0.16
Sterols [*μ*g/mL]	92.93	5.00	101.38	5.54	97.15	6.28	101.97	6.03

**Table 3:** Spearman's rank correlation coefficients [*r*_*s*_] between the total favourable effects of the emulsions as assessed with the multicriterial analysis (MCA) and the contents of selected group of compounds in the tested emulsions.

Compounds estimated in the tested emulsions	Spearman's rank correlation coefficient [*r*_*s*_]
Lipid-soluble antioxidants	0.8
Phenolics	0.8
Unsaturated fatty acids	−0.4
Squalene	0.8
Sterols	0.2

*r*_*s*_ ≤ 0.2: weak,

*r*_*s*_ ≤ 0.4: moderate,

*r*_*s*_ ≤ 0.8: strong,

*r*_*s*_ = 1.0: complete,

according to JP Guilford.

**Table 4:** Multicriterial analysis of tested emulsions in the aspect of their enhancement of fibroblasts activity in the culture. The results of six *in vitro* tests with emulsions added to the final concentration of 0.5% (v/v) of cell culture medium were analyzed. Cultures of V79 fibroblasts were carried out in the presence of tested emulsions for 48 h (test 1). For evaluation of antioxidative activity of the emulsions at the end of culture time cells were exposed to oxidative stress with H_2_O_2_ [100 *μ*M, 30 min, 4°C] (tests: 2–6). The multicriterial analysis was performed according to the method described in Section 2.

	Rating and ranking criteria			Tested emulsions			
	Test	Expected result	Index of importance	Linola	W92	W86	GT
(1)	Proliferation of V79 fibroblasts	Increase	0.2	0.123	5.714	13.604	1.235
(2)	Intracellular contents of ROS	Decrease	0.2	1.904	18.182	12.820	6.896
(3)	DNA contents in comets' head	Increase	0.2	0.188	0.144	0.766	0.268
(4)	Olive tail moment	Decrease	0.2	0.144	0.093	0.130	0.214
(5)	Frequency of apoptosis	Decrease	0.1	0.452	0.038	0.1618	0.022
(6)	Frequency of necrosis	Decrease	0.1	0.011	0.078	0.526	0.171
**Total** (**sum of the results in columns**)			**1.0**	**2.8225**	**24.2495**	**28.0078**	**8.8058**
